RETRACTED

# Human Sports Action and Ideological and PoliticalEvaluation by Lightweight Deep Learning Model

**DOI:** 10.1155/2022/5794914

**Published:** 2022-07-09

**Authors:** Mingqian Li, Jing Zhao

**Affiliations:** Xi'an International Studies University, Xi'an 710128, China

## Abstract

The purpose is to automatically and quickly analyze whether the rope skipping actions conform to the standards and give correct guidance and training plans. Firstly, aiming at the problem of motion analysis, a deep learning (DL) framework is proposed to obtain the coordinates of key points in rope skipping. The framework is based on the OpenPose method and uses the lightweight MobileNetV2 instead of the Visual Geometry Group (VGG) 19. Secondly, a multi-label classification model is proposed: attention long short-term memory-long short-term memory (ALSTM-LSTM), according to the algorithm adaptive method in the multi-label learning method. Finally, the validity of the model is verified. Through the analysis and comparison of simulation results, the results show that the average accuracy of the improved OpenPose method is 77.8%, an increase of 3.3%. The proposed ALSTM-LSTM model achieves 96.1% accuracy and 96.5% precision. After the feature extraction model VGG19 in the initial stage of OpenPose is replaced by the lightweight MobileNetV2, the pose estimation accuracy is improved, and the number of model parameters is reduced. Additionally, compared with other models, the performance of the ALSTM-LSTM model is improved in all aspects. This work effectively solves the problems of real-time and accurate analysis in human pose estimation (HPE). The simulation results show that the proposed DL model can effectively improve students' high school entrance examination performance.

## 1. Introduction

The extracurricular physical exercise of primary and secondary school students after school and holidays is gradually reduced. The rise of online teaching and online tutoring has squeezed the time for students to exercise after school. Artificial intelligence (AI), big data, cloud computing, and other technologies not only break through the limitations of traditional physical education (PE) classrooms due to factors such as space, time, and region but also provide a guarantee for the teaching feedback link in extracurricular PE teaching in schools. By changing the traditional interaction between teachers and students, teachers have redesigned PE teaching and adopted new learning evaluation methods so that PE teaching presents a new learning space and learning environment [1]. In recent years, vision-based human motion analysis technology has received extensive attention with the continuous development and application of computer technology and AI technology. At present, vision-based human motion analysis is still a major challenge in the field of computer vision, mainly involving pattern recognition, image processing, virtual reality (VR), and other disciplines. It has broad application prospects in the fields of human-computer interaction (HCI), rehabilitation therapy, and sports training [2, 3].

RETRACTED

Computer vision has been widely used in sports training and other related fields, including motion type recognition and activity recognition, athlete tracking, and human pose estimation (HPE). The core problem of motion analysis is HPE. This is an important topic in the field of computer vision. The task of HPE is to identify the human body through computer image processing algorithms and determine the joint positions of the human body (such as eyes, nose, shoulders, wrists, and so on) [4–6]. The application of HPE involves human behavior understanding, HCI, health monitoring, motion capture, and other fields. Nadeem et al. [7] proposed a new method for automatic HPE. The method intelligently recognizes human behavior by utilizing salient contour detection, robust body part models and multi-dimensional cues from full-body contours, and the maximum entropy Markov model (MEMM). Firstly, the image is preprocessed and noise is removed to obtain robust contours. Then, the body part model is used to extract 12 key body parts. These key body parts are further optimized to help generate multi-dimensional cues. Finally, MEMM is used to process these optimization modes further, using a cross-validation scheme that omits one term. Better body part detection and higher identification accuracy are achieved on four benchmark datasets, with results superior to existing well-known statistical latest methods. Cui and Dahnoun [8] proposed an HPE system based on millimeter-wave radar. The system detects persons with arbitrary poses at close range (within two meters) in indoor environments and estimates poses by locating key joints. Two-millimeter wave radars were used to capture the scene, and a neural network model was used to estimate the pose. The neural network model consists of a part detector that estimates the position of the subject's joints and a spatial model that learns the correlations between the joints. A time-dependent step is introduced in real-time operation to refine the estimation further. The system is able to provide accurate HPE in real-time at 20 frames per second, with an average localization error of 12.2 cm and an average accuracy of 71.3%. Wu et al. [9] proposed a model in which multiple subnets are connected in parallel on the high-resolution main net. It maintains the network structure of high-resolution heat maps throughout the operation. The structure is applied to the human body key point vector field network, which improves the accuracy and operation speed of human body gesture recognition. Experimental results show that the proposed network outperforms existing mainstream research by 3%-4%. To sum up, the deep learning (DL) model is widely used in the field of computer science. Applying it to fields such as safety monitoring, health assessment, and HCI search can help recognize human actions according to human joints using sensors. For example, convolutional neural network (CNN) can be used for feature extraction, and multi-layer perceptron can be used as the standard for subsequent classification. These findings show that CNN-based supervised learning is very effective.

RETRACTED

The key to improving the performance of the rope skipping test is to automatically and quickly analyze whether the rope skipping action meets the standards and give correct guidance and training plans. The existing HPE algorithms based on computer vision have high complexity, poor robustness, and complex computation. Additionally, due to the lack of professional human action analysts, the research on human action analysis and sports quality evaluation needs to be further explored. The innovation of this work is that the coordinates of the key points in the rope skipping process are obtained through the two-dimensional (2D) HPE algorithm. The coordinates are preprocessed to obtain a robust data sequence. A multi-label classification model is proposed: attention long short-term memory-long short-term memory (ALSTM-LSTM). The proposed model can effectively solve the problems of real-time analysis and accurate analysis. The results show that the ALSTM-LSTM model can improve students' high school entrance examination scores.

## 2. Materials and Methods

### 2.1. Smart Sports

The basic task of smart sports is to obtain the pose changes of the human body through the equipment and analyze and guide the attitude [10, 11]. In recent years, measurement technologies such as accelerometers, gyroscopes, and magnetometers have emerged. However, these technologies rely heavily on specialized equipment, which is very expensive. Professional competitive sports training mostly adopts traditional methods, and the training requirements are very high. It needs to invest extensive human and financial resources to make professional sports training smart [12]. Emerging technologies such as AI and big data have been widely used in sports evaluation and guidance. The sports data acquisition and analysis system utilizes wearable devices to capture and record students' actions during physical exercise and further evaluates their actions against specific standards. Based on virtual reality (VR) technology, a more in-depth experimental study on the PE teaching platform simulates human action scenes. With the in-depth development of deep neural networks and hardware technology, AI technology based on DL has shown relatively good results in HPE [13, 14]. The HPE method based on DL can predict the data information of human skeleton points from each video frame and finally regenerate the human skeleton.

RETRACTED

### 2.2. 2D Human Pose Estimation Based on OpenPose

The OpenPose Estimation Project is an open-source library based on convolutional neural network (CNN) and supervised learning. It is regarded as a skeleton point and skeleton detector, which can predict human facial key points, limb skeleton points, hand joint points, and other parts. It shows good robustness in the pose estimation of one or more people. The input of OpenPose can realize pictures, videos, or real-time cameras as input and output the position and coordinate information of the joint points of the human body through OpenPose estimation [15]. The basic principle of OpenPose is to build a CNN in stages and then output the prediction confidence heat map of the skeleton points after predicting the human skeleton points in the image. Additionally, it also predicts the affinity field between bones. The affinity field is the basis for connecting the skeleton and participates in the next stage of skeleton point prediction, improving the speed and accuracy of the model [16, 17]. The OpenPose processing flow is shown in Figure 1. It learns using nonparametric representations through partial affinity fields, associating body parts with individuals in images, giving a bottom-up representation of the distribution of limb associations.

In Figure 1, in order to obtain the key point coordinate information of the human body in the human body pose estimation based on OpenPose, it is necessary to use the Gaussian modeling method to obtain the confidence map of the key point position. A confidence map represents key points. The values in the confidence map represent the probability of a certain key point location [18, 19]. Confidence maps of key point locations are shown in equations (1) and (2):

(1) $$\begin{array}{c} S_{j,k}=\exp\left(-\frac{{\left\|p-x_{j,k}\right\|}_{2}^{2}}{\delta^{2}}\right), \end{array}$$

(2) $$\begin{array}{c} S_{j}\left(p\right)=\max\underset{k}{S_{j,k}}\left(p\right), \end{array}$$

where *S*_*j,k*_ represents the confidence map of the individual produced by each individual *k*; *k* represents the *k*-th individual in the image; *j* represents the *j*-th joint point of the individual; *p* represents the coordinates of the predicted individual in the image; *δ* represents a minimum value, which can ensure certain feasibility in the training process of the model; and *x*_*j,k*_ represents the real coordinate position of the *j*-th joint point of the *k*-th individual.

RETRACTED

### 2.3. Multi-Label Classification Method

In practical applications, a person's body movements need to be analyzed in many aspects, and there are often multiple labels in one frame of the image. In the multi-label classification problem, there is a certain dependency or mutual exclusion between labels. In multi-label classification tasks, the relationship between categories is very complex due to the large number of labels. Therefore, multi-label classification is more complex than single-label classification [20, 21]. According to the source of algorithm design ideas, there are two types of methods for multi-label classification problems: problem transformation methods and algorithm adaptation methods, as shown in Figure 2. Problem conversion-based methods usually transform multi-label classification problems into other learning scenarios. As shown in Figure 2, the multi-label learning method can be divided into two categories: problem conversion method and algorithm adaptation method. They are represented by the left block diagram and the right frame diagram, respectively. The problem conversion-based method adapts the current popular algorithm in the classification process to process multi-label data, such as the adaptive DL algorithm and recurrent neural network (RNN), to apply them to many label classification tasks [22].

### 2.4. Action Analysis Algorithm in Rope Skipping Scenario

#### 2.4.1. MobileNetV2 Framework

The lightweight network model is to make the model run in a shorter time and consume fewer resources while maintaining accuracy. When acquiring the human pose, the OpenPose network model first sends the image frame to the Visual Geometry Group (VGG) 19 to obtain a collection of image feature maps. However, VGG19 is computationally expensive. Also, it produces a lot of parameters during training. Therefore, the occupied memory is also large [23]. However, the model trained by the MobileNetV2 network is small, fast in speed, and has high accuracy. Therefore, when extracting image feature maps, the original OpenPose method is changed to MobileNetV2.

The MobileNetV2 network is improved based on MobileNet. An inverted residual structure is added to MobileNetV2. The inverted residual structure first maps low-dimensional features to high-dimensional features, then uses depth-wise separable convolution to perform convolution operations, and then uses a linear convolution to map them to low-dimensional features. In order to make the model have better expressiveness in the calculation process, the nonlinear transformation in MobileNet is removed in the MobileNetV2 network. Meanwhile, a linear bottleneck is also introduced in MobileNetV2 [24]. In MobileNetV2, it is believed that the nonlinear activation function of each layer in the neural network will bring two problems to the network: the first is that after the ReLU activation function, the input data and output data are linearly transformed, and the obtained output result is nonzero. The other is that if the integrity of the interest manifold in the activation space is high, the problem of space collapse will occur after the ReLU activation function. Then, the architecture of MobileNetV2 is analyzed by referring to relevant literature [25]. The structure of MobileNetV2 is unfolded in Table 1. Here, — indicates that the structure parameter value of this network layer does not exist. The network first uses full convolution as 32 convolution kernels and then uses 19 inverse residual structures with linear bottlenecks. Such low precision computation has stronger robustness. Further, *t* represents the “spread” factor: the channel spread factor of the inverse residual network. *c* stands for the number of output channels. *n* refers to the number of repetitions. *n* denotes the step length.

RETRACTED

#### 2.4.2. ALSTM-LSTM Network Framework

DL has strong learning properties and the ability to analyze rules between data. The use of this technology is beneficial to promote the development of data visualization and classification management. DL works by incrementally approximating complex functions by learning from deep nonlinear networks. Its model structure learning is more in-depth compared with the traditional artificial neural network. There are many nodes in the hidden layer that emphasize feature learning of the data. DL is to transform the feature representation of samples in the original space into a new feature space, simplify the classification and prediction of data, learn in fewer samples, and express complex functions with fewer parameters. This reduces the difficulty of setting and adjusting model parameters, contains more hidden layers than traditional shallow neural networks, and can learn more rich sample features. Additionally, its simulation performance is also better [26]. The long short-term memory network (LSTM) is essentially derived from the RNN. LSTM is a state unit added to the RNN. Its function is to save the previously input information, and a gating mechanism with three gates is also designed, and the activation function and excitation function are set in the structure of each gate. In general, the tanh function is chosen as the activation function for the input and output of the memory cell. The sigmoid function is used as the activation function of the gate structure [27].

RETRACTED

The human pose analysis problem during jumping is transformed into a multi-label classification problem with a temporal relationship. LSTM can play a role in global processing and storage units so that LSTM can maintain relatively good performance in time series. Attention is a global processing method. Therefore, attention is applied to LSTM and combined with a single LSTM for multi-label classification, which is the ALSTM-LSTM method. The specific network framework is shown in Figure 3.

In Figure 3, the ALSTM-LSTM network includes five layers: input, batch normalization, ALSTM-LSTM, connection, and sigmoid layer. Additionally, a batch normalization layer is added before the LSTM and ALSTM layers. The study is a multi-label classification problem. According to the multi-label algorithm transformation method, the activation function of the last layer of the ALSTM-LSTM model is set to the sigmoid function, and the loss function selects the binary cross-entropy.

In the two branches of OpenPose, one branch is used to predict the confidence of key points, and the other branch is used to predict the affinity field between two key points. The overall loss is the sum of each stage, as shown in the following equation:

(3) $$\begin{array}{c} f=\sum_{t=1}^{T}\left(f_{S}^{t}+f_{L}^{t}\right), \end{array}$$

where *S* represents the confidence of the key point; *L* represents the affinity field between two key points; *f*_*S*_^*t*^ represents the loss in the confidence stage of predicting key points; and *f*_*L*_^*t*^ represents the loss in this stage of predicting the affinity field between two key points.

### 2.5. Dataset and Experimental Environment Settings

#### 2.5.1. Dataset

The dataset used in the experiment is the Max Planck Institute for Informatics (MPII) dataset. The MPII human pose dataset is a benchmark for estimation. The dataset includes 25,000 annotated images of more than 40,000 people and contains 410 regularly performed human activities with corresponding labels. These images are pulled from YouTube. The test set includes annotations for body part occlusion, 3D torso, and head orientation. The MPII dataset is used to train the network model and detect key point coordinates of the head, shoulders, wrists, hips, knees, and ankles.

In addition, many countries and regions include one-minute hopping in the middle school entrance examination. The rope skipping dataset used is from an experimental high school. In different scenarios, different mobile phones are used to shoot videos from the front and store them in MP4 format. Different mobile phones take images with different pixels. At present, 200 middle school students have one-minute rope skipping video streaming data collected. The age group of students is 11–15 years old. The distribution of male and female students among the 200 students collected is shown in Figure 4.

RETRACTED

In Figure 4, professionals get data labels by analyzing videos and labeling them by time segments. The labels of the data are set to six labels, namely, the body is kept upright, the left wrist is rocked, the left arm is tightened with the body, the right wrist is shaken, the right arm is tightened with the body, and the left and right arms are kept horizontal, as shown in Figure 5. The selection of these labels is based on the skipping skills of the mid-admission exam.

In Figure 5, because the captured images are the same, the dataset needs to be preprocessed. Preprocessing of video frames includes setting video frames of different sizes to the same size. The video height and width are set to 530 pix and 460 pix, respectively. The basic information of each skipping object, including name, age, gender, height, and weight, is recorded and saved. The key point detection method is used to obtain the nose, neck, right shoulder, right elbow, right wrist, left shoulder, left elbow, left wrist, right hip, right knee, right ankle, left hip, and left knee—the coordinate positions of the 14 joint points of the left ankle. The obtained 14 key point coordinates define a Cartesian coordinate system with the center of gravity of the triangle formed by the three points of the left hip, right hip, and neck as the origin. The coordinate matrix obtained in each frame is accumulated to obtain the cumulative coordinate matrix of each video.

#### 2.5.2. Setting of the Experimental Environment

In the process of pose estimation and skipping action analysis, the code is written in PyCharm and Jupyter Notebook. Intel Core i7-8700K, 3.70 GHz, is used. Memory is 32G; GPU is GTX 1080Ti. In LSTM, units are set to 64 and batch size is set to 100. In order to choose an appropriate sliding window length, the sliding window length is set to 10 frames and 15 frames, the cumulative coordinates are set to 20 frames, and the step size is set to 30% data overlap.

The evaluation indicators of human key point detection are object key point similarity (OKS), average precision (AP), and mean average precision (MAP). Among them, OKS is to calculate the similarity between the real value and the predicted human key points, as shown in the following equation:

(4) $$\begin{array}{c} {\text{OKS}}_{p}=\frac{\sum_{i}\exp\left\{-d_{p^{2}}^{2}/2S_{p}^{2}\sigma_{i}^{2}\right\}\delta \left(vp^{i}>0\right)}{\sum_{i}\delta \left(vp^{i}>0\right)}, \end{array}$$

where *p* represents the id of a person in the ground truth; pi represents the key point id of a person; *vp*^*i*^ = 0 means that key points are not labeled; *vp*^*i*^ = 1 means that the key points are occluded but marked; *vp*^*i*^ = 2 means that the key points are unobstructed and marked; *S*_*p*_ is the square root of the size of the area occupied by the person; *σ*_*i*_ represents the normalization factor of the *i*-th bone point; and *δ*(.) is 1 when the condition holds; it is 0 otherwise.

RETRACTED

Common evaluation indicators for multi-label classification are accuracy, *F*1-score, precision, and recall. The calculation of each indicator is shown in equations (5)–(8):

(5) $$\begin{array}{c} \text{precision}=\frac{\text{TP}}{\text{TP}+\text{FP}}, \end{array}$$

(6) $$\begin{array}{c} \text{recall}=\frac{\text{TP}}{\text{TP}+\text{FN}}, \end{array}$$

(7) $$\begin{array}{c} \text{accuracy}=\frac{\text{TP}+\text{TN}}{\text{TP}+\text{FP}+\text{TN}+\text{FN}}, \end{array}$$

(8) $$\begin{array}{c} F1=\frac{2\text{TP}}{2\text{TP}+\text{FP}+\text{FN}}, \end{array}$$

where true positives (TP) are positive samples that are correctly identified as positive samples; true negatives (TN) are negative samples that are correctly identified as negative samples; false positives (FP) are negative samples that are incorrectly identified as positive samples; and false negatives (FN) are positive samples that are misidentified as negative samples.

## 3. Results and Discussion

### 3.1. Analysis of the Experimental Results of Attitude Estimation

In order to improve the accuracy and efficiency of pose estimation, the feature extraction model VGG19 in the initial stage of OpenPose is replaced by a lightweight network model MobileNetV2. Weights and penalties are introduced into the final loss function. The experimental results on the MPII dataset are shown in Figure 6.

In Figure 6, the MAP of OpenPose is 74.5%. The MAP of the improved OpenPose method is 77.8%, and the MAP is improved by 3.3%. After replacing the feature extraction model VGG19 in the initial stage of OpenPose with the lightweight network model MobileNetV2, the pose estimation accuracy has been improved, and the total number of parameters of the model has been reduced. Therefore, the improved OpenPose model structure can meet the experimental requirements.

### 3.2. Analysis of the Experimental Results of Multi-Label Classification of Rope Skipping

Since the rope skipping process is a long-term sequence analysis process, it is necessary to segment the data through a sliding window. In this experiment, three groups of 10-frame cumulative coordinates, 15-frame cumulative coordinates, and 20-frame cumulative coordinates are set up for analysis to find the appropriate sliding window length. The step size is set to 30% data overlap. The specific experimental results are shown in Figure 7.

RETRACTED

In Figure 7, when the sliding window length is 10, the accuracy of ALSTM-LSTM is 85.36%, and the *F*1 value is 83.13%. When the sliding window length is 15, the accuracy of ALSTM-LSTM is 89.55%, and the *F*1 value is 88.75%. When the sliding window length is 20, the accuracy of ALSTM-LSTM is 87.77%, and the *F*1 value is 86.43%. Therefore, ALSTM-LSTM performs best when the sliding window length is 15.

Support vector machine (SVM) is a linear classifier model defined in feature space. This algorithm can effectively help optimize quadratic programming. The performance of the proposed ALSTM-LSTM model and SVM model is compared to further verify and optimize the proposed model. The results are given in Figure 8.

In Figure 8, in the multi-label classification problem of skipping action analysis, the proposed ALSTM-LSTM model achieved an accuracy of 96.1%, precision of 96.5%, recall of 95%, and *F*1 value of 95.7%. DL models outperform traditional machine learning algorithms. In the rope skipping action analysis, the ALSTM-LSTM architecture provides the best performance on all metrics, and the SVM has the worst performance.

To sum up, this work studies the recognition and evaluation of 2D human poses based on OpenPose and designs. It analyzes the ALSTM-LSTM network framework by combining the multi-label classification method. The results show that the MAP of the OpenPose method before and after optimization is 74.5% and 77.8%, respectively, improved by 3.3%. After replacing the feature extraction model VGG19 in the initial stage of OpenPose with the lightweight network model MobileNetV2, the pose estimation accuracy is improved, and the model parameters are reduced. Some other scholars' research results are cited below. Ding et al. [28] researched HPE based on multi-feature and rule learning and proposed a new algorithm based on multi-feature and rule learning. The research results showed that feature fusion at the granularity level could reduce the dimension and sparsity of feature sets. Zhang and Callaghan [29] conducted real-time HPE based on an adaptive hybrid classifier. The pose-based adaptive signal segmentation algorithm was combined with a multi-layer perceptron classifier, and various voting methods were combined. A sensor calibration algorithm based on software was designed. The results showed that the adaptive hybrid classifier could improve the accuracy of real-time HPE. To sum up, the proposed improved HPE algorithm can improve the recognition accuracy of the system for human actions.

RETRACTED

## 4. Conclusion

The HPE task is to recognize human body through computer image processing algorithm. The application of HPE involves human behavior understanding, HCI, health monitoring, motion capture, and other fields. Following a review of smart sports, the research is based on the lightweight DL model. OpenPose is used to design and evaluate human poses. The multi-label classification algorithm is used to design the architecture of MobileNetV2. The research content is based on the pose analysis in the scene of shaking feet and skipping rope in the high school entrance examination. Combined with the characteristics of the research scene, the HPE model based on OpenPose network and the multilabel classification network structure are introduced. In order to improve the efficiency and accuracy of pose analysis, OpenPose is improved based on the lightweight network MobileNetV2. Then, the ALSTM-LSTM model is proposed to analyze whether the body actions are standardized during rope skipping. The results show that MAP of the OpenPose method based on MobileNetV2 is improved by 3.3% compared to the standard OpenPose method. In the multi-label classification problem of skipping action analysis, the ALSTM-LSTM model achieves 96.1% accuracy, 96.5% precision, 95% recall, and 95.7% *F*1 value. The ALSTM-LSTM architecture provides the best performance on all metrics for skipping action analysis. The disadvantage is that in the physics test of the middle school entrance examination, rope skipping is the research object, but the research method is not limited to this scenario. In the future work, ALSTM-LSTM architecture will collect more rope skipping videos from different scenes to provide stronger data support for subsequent action analysis. The research has practical reference value for applying lightweight DL model in HPE.

## Figures and Tables

**Figure 1:** Flow of OpenPose processing.

**Figure 2:** Multi-label learning method.

**Figure 3:** Network framework of ALSTM-LSTM.

**Figure 4:** Distribution of the rope skipping dataset.

**Figure 5:** Marker names for body movements.

**Figure 6:** Experimental results of the MPII dataset.

**Figure 7:** Sliding window selection.

**Figure 8:** Comparison of the ALSTM-LSTM model with other models.

**Table 1:** Structure of MobileNetV2 network.

Input	Operator	*t*	*c*	*n*	*s*
224^2^ × 3	Conv2d	—	32	1	2
112^2^ × 32	Bottleneck	1	16	1	1
112^2^ × 16	Bottleneck	6	24	2	2
56^2^ × 24	Bottleneck	6	32	3	2
28^2^ × 32	Bottleneck	6	64	4	2
14^2^ × 64	Bottleneck	6	96	3	1
14^2^ × 96	Bottleneck	6	160	3	2
7^2^ × 160	Bottleneck	6	320	1	1
7^2^ × 320	Conv2d 1 × 1	—	1280	1	1
7^2^ × 1280	Avg pool 7 × 7	—	—	1	—
1 × 1 × *k*	Conv2d 1 × 1	—	*k*	—	—

RETRACTED

## Data Availability

The data used to support the findings of this study are available from the corresponding author upon request.
